The article "Analysis of the B2M Expression in Colon Adenocarcinoma and Its Correlation with Patient Prognosis" was retracted in 2023. Reasons: suspected computer-generated content; unreliable results or conclusions; lack of ethics approval or compliance; missing or withdrawn patient consent.

# Analysis of the B2M Expression in Colon Adenocarcinoma and Its Correlation with Patient Prognosis

**DOI:** 10.1155/2022/7264503

**Published:** 2022-08-09

**Authors:** Hailian Lin, Kelang Wang, Kebing Zou, Yuanyuan Wang, Gen xiang Que, Xuefeng Yang, Mengdan Liao

**Affiliations:** ^1^Hunan Provincial Clinical Research Center for Metabolic Associated Fatty Liver Disease, the Affiliated Nanhua Hospital, Hengyang Medical School, University of South China, Hengyang 421002, Hunan, China; ^2^The Affiliated Nanhua Hospital, Department of Gastroenterology, Hengyang Medical School, University of South China, Hengyang 421002, Hunan, China; ^3^The Affiliated Nanhua Hospital, Department of General Practice, Hengyang Medical School, University of South China, Hengyang 421002, Hunan, China; ^4^The Affiliated Nanhua Hospital, Department of Nephrology, Hengyang Medical School, University of South China, Hengyang 421002, Hunan, China

## Abstract

Colon adenocarcinoma (COAD) is one of the most common malignant tumors in clinics. It is often found at an advanced stage, with high incidence and poor prognosis; early diagnosis is difficult and treatment methods are limited. In order to find new methods for diagnosis and treatment of COAD, people pay more and more attention to the discovery and functional research of new oncogenes and tumor suppressor genes of COAD. *β*2-microglobulin (B2M) plays different physiological and pathological roles in tumor cells and nontumor cells. At present, there is no public report on the expression of B2M in COAD. In this study, the expression of B2M mRNA in COAD tissues was compared with that in normal tissues. The relationship between the expression of B2M mRNA and the stage, histological subtype, lymph node metastasis, TP53 mutation, and survival time of COAD was discussed. It was found that B2M is a potential tumor suppressor gene in COAD. The decreased expression of B2M after mutation can cause immune escape of COAD cells, thus affecting the therapeutic effect and prognosis. This study provides a new idea for the prevention and treatment of COAD.

## 1. Introduction

Colon adenocarcinoma (COAD) is one of the most common malignant tumors in the clinics. It is often found at an advanced stage, with high incidence and poor prognosis, and early diagnosis is difficult and treatment methods are limited. In order to find new methods for diagnosis and treatment of COAD, people pay more and more attention to the discovery and functional research of new oncogenes and tumor suppressor genes of COAD.

*β*2-microglobulin (B2M) is a serum protein composed of 119 amino acids with a size of 12 kDa [1]. B2M is expressed in all nucleated cells and is an important subunit of major histocompatibility complex (MHC) class I. It plays different physiological and pathological roles in tumor cells and nontumor cells, especially performing important biological functions in immune monitoring [2]. A large number of studies have found that serum B2M protein is closely related to infection [3, 4], cardiovascular and cerebrovascular diseases [5–7], inflammatory bowel disease [8], kidney injury [9], blood system diseases [10–12], amyloidosis [13, 14], and aging-related diseases [15]. At present, there is no public report on the expression of B2M in COAD. The purpose of this study is to use the TCGA database to analyze the difference of the B2M gene mRNA expression between colon cancer tissues and normal colon tissues and its correlation with the survival prognosis of patients, so as to provide new diagnostic markers and therapeutic targets for colon adenocarcinoma.

The article "Analysis of the B2M Expression in Colon Adenocarcinoma and Its Correlation with Patient Prognosis" was retracted in 2023. Reasons: suspected computer-generated content; unreliable results or conclusions; lack of ethics approval or compliance; missing or withdrawn patient consent.

## 2. Methods

### 2.1. Experimental Methods

The experimental methods are as follows:

1. TCGA database was used to analyze the expression of B2M mRNA in pan-cancer tissues and corresponding normal tissues.
2. UALCAN (https://ualcan.path.uab.edu/index.html) is an effective online cancer data analysis and mining website based on relevant cancer data in TCGA database. We accessed the TCGA database through the UALCAN website [16] to analyze the expression of B2M mRNA in pan-cancer tissues and corresponding normal tissues.
3. TCGA database was used to analyze the difference of the B2M mRNA expression between colon adenocarcinoma tissues and normal colon tissues.
4. We accessed the TCGA database through the UALCAN website [16], from which we downloaded 286 colon cancer tissue samples and 41 paracancer normal tissue samples to analyze the difference of the B2M mRNA expression between colon cancer tissues and adjacent normal tissues.
5. TCGA database was used to analyze the difference of methylation level of a B2M gene promoter between colon adenocarcinoma tissues and normal colon tissues.
6. We accessed the TCGA database through the UALCAN website [16] to analyze the difference of methylation level of the B2M gene promoter between colon cancer tissues and adjacent normal tissues.
7. TCGA database was used to analyze the relationship between B2M mRNA expression and colon cancer stage.
8. According to the latest TNM staging of malignant tumor, colon cancer can be divided into four stages according to the severity: Stage 1: The primary tumor is only confined to the mucosa or submucosa, and there is no tumor lymph gland metastasis or distant metastasis. Stage 2: The primary tumor invaded the muscular layer of intestinal wall, but there is no tumor lymph gland metastasis or distant metastasis. Stage 3: No matter the depth of primary tumor invasion, regional lymph node metastasis has occurred, but there is no distant metastasis. Stage 4: The tumor had distant metastasis, such as liver, lung, bone, and brain metastasis, peritoneal implantation metastasis, and distant lymph node metastasis(such as supraclavicular lymph node metastasis) [17]. We accessed the TCGA database through the UALCAN website [16] to analyze the relationship between the expression of B2M mRNA and the stage of colon cancer.
9. TCGA database was used to analyze the relationship between B2M mRNA expression and histological subtypes of colon cancer.
10. The histological types of colon cancer can be divided into the following types: (1) Nonspecific adenocarcinoma. (2) Special types of adenocarcinoma, including mucinous adenocarcinoma, medullary carcinoma, serrated adenocarcinoma, signet-ring cell adenocarcinoma, cribriform acne adenocarcinoma, and micropapillary adenocarcinoma. (3) Squamous cell carcinoma. (4) Adenosquamous carcinoma. (5) Spindle cell carcinoma/sarcomatoid carcinoma. (6) Undifferentiated carcinoma. (7) Other special types of colon cancer. (8) Type undetermined colon cancer [18]. We accessed the TCGA database through UALCAN website [16] and mainly analyzed the differences of the B2M mRNA expression between adenocarcinoma and mucinous adenocarcinoma.
11. TCGA database was used to analyze the relationship between the B2M mRNA expression and lymph node metastasis.
12. The status of lymph node metastasis was divided into four grades: N0: no regional lymph node metastasis; N1:1∼3 axillary lymph nodes metastasis; N2:4∼9 axillary lymph nodes metastasis; N3:more than 10 axillary lymph nodes metastasis. We accessed the TCGA database through the UALCAN website [16] to analyze the relationship between the B2M mRNA expression and lymph node metastasis.
13. TCGA database was used to analyze the relationship between the B2M mRNA expression and TP53 mutation status.
14. We accessed the TCGA database through the UALCAN website [16] to analyze the relationship between the B2M mRNA expression and TP53 mutation status.
15. TCGA database was used to analyze the relationship between the B2M mRNA expression and gender, age, weight, and race of patients with colon cancer.
16. We accessed the TCGA database through the UALCAN website [16] to analyze the relationship between the B2M mRNA expression and gender, age, weight, and race of patients with colon adenocarcinoma.
17. TCGA database was used to analyze the relationship between the expression level of B2M mRNA in colon adenocarcinoma. tissues and the survival time of patients.
18. TCGA database was used to analyze the genes related to the B2M gene expression in patients with colon adenocarcinoma.
19. We accessed the TCGA database through the UALCAN website [16] to analyze the genes related to the B2M gene expression in colon adenocarcinoma patients.

The article "Analysis of the B2M Expression in Colon Adenocarcinoma and Its Correlation with Patient Prognosis" was retracted in 2023. Reasons: suspected computer-generated content; unreliable results or conclusions; lack of ethics approval or compliance; missing or withdrawn patient consent.

### 2.2. Statistical Analysis

Wilcoxon assay was used to analyze the expression levels of B2M mRNA in colon cancer tissues and normal colon tissues. Kaplan–Meier analysis was used to compare the survival time of the B2M mRNA high expression group and low expression group. Log-ranch test was used to calculate the *p* value, *P* < 0.05 indicates statistical significance. All statistical analyses were performed using R (version x64 3.5.1).

## 3. Results

### 3.1. Clinical Characteristics of 286 Patients with Colon Cancer in the TCGA Database

We downloaded the clinical data of 286 patients with colon cancer from TCGA database, including patients' gender, age, weight, race, clinical stage, and histological subtype. After excluding the samples with incomplete clinical data, in the categories of gender, age, weight, clinical stage, and histological subtype, only 283, 283, 210, 274, and 280 samples were left to participate in the statistics; the clinical characteristics are shown in Table 1.

### 3.2. The Expression of B2M mRNA in Pan-Cancer Tissues and Corresponding Normal Tissues

The expression of B2M mRNA in pan-cancer tissues and corresponding normal tissues is shown in Figure 1. It can be seen that the expression of B2M mRNA is increased in most tumors, such as BRCA (*p*=1.604910*E* − 03), CHOL (*p*=7.43370000000354*E* − 07), ESCA (*p*=1.63501000000066*E* − 05), GBM (*p*=1.62447832963153*E* − 12), HNSC (*p*=1.62458935193399*E* − 12), KICH (*p*=3.87309999627661*E* − 08), KIRC (*p* < 1*E* − 12), KIRP (*p*=1.5612000003884*E* − 07), PCPG (*p*=<1*E* − 12), THCA (*p*=3.298400*E* − 03). In a few tumors, the expression of B2M mRNA was decreased, such as COAD (*p* < 1*E* − 12), LUAD (*p*=1.62436730732907*E* − 12), LUSC (*p*=1.62458935193399*E* − 12), PRAD (*p*=1.757730*E* − 02), and READ (*p*=1.82229999978745*E* − 08). There was no statistically significant differences in the expression of other tumors in Figure 1.

### 3.3. The Expression of B2M mRNA in Colon Adenocarcinoma Tissues Was Significantly Lower Than That in Normal Colon Tissues

We downloaded 41 samples of normal tissues adjacent to cancer and 286 samples of colon cancer from the TCGA database. It can be seen that the expression of B2M mRNA in colon adenocarcinoma tissues was significantly lower than that in adjacent normal tissues (*p* < 1*E* − 12) (Figure 2).

### 3.4. The Methylation Level of a B2M Gene Promoter in Colon Adenocarcinoma Tissues Was Lower Than That in Normal Colon Tissues

The results of TCGA database analysis showed that the methylation level of B2M gene promoter in colon cancer tissues was lower than that in normal colon tissues, and the difference was statistically significant (*p*=1.959910*E* − 03) (Figure 3).

*β* values indicate DNA methylation levels from 0 (unmethylated) to 1 (fully methylated). Different *β* value represents hypermethylation (*β* values: 0.7–0.5) or hypomethylation (*β* values: 0.3–0.25).

The article "Analysis of the B2M Expression in Colon Adenocarcinoma and Its Correlation with Patient Prognosis" was retracted in 2023. Reasons: suspected computer-generated content; unreliable results or conclusions; lack of ethics approval or compliance; missing or withdrawn patient consent.

### 3.5. The Expression Level of B2M mRNA Was Correlated with the Stage of Colon Adenocarcinoma

The results of TCGA database analysis showed that the expression level of B2M mRNA was correlated with the stage of colon cancer. The difference of B2M mRNA expression between stage I and stage IV, and between stage II and stage IV was statistically significant. The higher the stage of colon cancer, the lower the expression of B2M mRNA (normal-vs-stage1: *p*=2.42909999892404*E* − 08; normal-vs-stage2: *p*=2.26879626197274*E* − 11; normal-vs-stage3: *p*=3.46889961200247*E* − 10; normal-vs-stage4: *p*=8.27404811332144*E* − 12; stage1-vs-stage4: *p*=1.609760*E* − 02; stage2-vs-stage4: *p*=3.202300*E* − 03) (Figure 4).

### 3.6. The Expression of B2M mRNA Was Correlated with Histological Subtypes of Colon Adenocarcinoma

The results of TCGA database analysis showed that the expression level of B2M mRNA was correlated with the histological subtypes of colon cancer, and the expression level of B2M mRNA in adenocarcinoma was lower than that in mucinous adenocarcinoma, and the difference was statistically significant (normal-vs-adenocarcinoma: *p*=1.34860012046545*E* − 10; normal-vs-mucinous-adenocarcinoma: *p*=2.019200*E* − 04; adenocarcinoma-vs-mucinous-adenocarcinoma: *p*=3.139800*E* − 02) (Figure 5).

### 3.7. The Expression of B2M mRNA Was Not Correlated with Lymph Node Metastasis

TCGA database analysis showed that B2M mRNA expression was not associated with lymph node metastasis (normal-vs-N0: *p*=1.79600001537494*E* − 09; normal-vs-N1: *p*=2.08109973698356*E* − 10; normal-vs-N2: *p*=1.10179976253733*E* − 10) (Figure 6).

### 3.8. B2M mRNA Expression Was Correlated with the TP53 Mutation Status

The results of TCGA database analysis showed that the expression level of B2M mRNA in colon adenocarcinoma tissues was correlated with the TP53 mutation status, and the expression level of B2M mRNA in TP53 mutated colon cancer tissues was lower than that in nonmutated colon adenocarcinoma tissues (normal-vs-tp53-mutant: *p*=5.69789770921147*E* − 11; normal-vs-tp53-nonmutant: *p*=6.83500001041892*E* − 09; tp53-mutant-vs-tp53-nonmutant: *p*=8.608400*E* − 04) (Figure 7).

### 3.9. The Expression Level of B2M mRNA Was Not Related to Gender, Age, and Weight of Patients with Colon Adenocarcinoma but Was Related to Race

The results of TCGA database analysis showed that the expression level of B2M mRNA in colon cancer tissues was not related to gender (normal-vs-male: *p*=2.39808173319034*E* − 14; normal-vs-female: *p*=1.88882243179478*E* − 12) (figure 8), age (normal-vs-age (21–40yrs): *p*=6.42129999999241*E* − 05; normal-vs-age (41–60yrs): *p*=4.14730028097665*E* − 10; normal-vs-age (61–80yrs): *p*=1.69331215715829*E* − 12; normal-vs-age (81–100yrs): *p*=4.07770000000474*E* − 05) (figure 9), and weight (normal-vs-normal weight: *p*=1.24109611476797*E* − 11; normal-vs-extreme weight: *p*=8.13670020249901*E* − 10; normal-vs-obese: *p*=2.16919999740384*E* − 08; normal-vs-extreme obese: *p*=5.75699999999513*E* − 05) (Figure 10), but was related to race, and the expression level of B2M mRNA in colorectal cancer tissues of African Americans was lower than that of Caucasians and Asians (normal-vs-Caucasian: *p*=1.74682490694522*E* − 12; normal-vs-African–American: *p*=1.28740351712509*E* − 11; normal-vs-Asian: *p*=5.421000*E* − 03; Caucasian-vs-African–American: *p*=1.956210*E* − 02; African–American-vs-Asian: *p*=2.269800*E* − 02) (Figure 11).

The article "Analysis of the B2M Expression in Colon Adenocarcinoma and Its Correlation with Patient Prognosis" was retracted in 2023. Reasons: suspected computer-generated content; unreliable results or conclusions; lack of ethics approval or compliance; missing or withdrawn patient consent.

### 3.10. The Expression of B2M mRNA Was Not Associated with the Survival of Patients with Colon Adenocarcinoma

Analysis of TCGA database showed that the expression of B2M mRNA was not associated with the survival of patients with colon cancer(*p*=0.75) (Figure 12).

### 3.11. Genes Related to the B2M Gene Expression in Patients with Colon Adenocarcinoma

Using TCGA database, we analyzed the top 25 genes positively correlated (Figure 13) and negatively correlated with B2M gene expression in colon adenocarcinoma patients (Figure 14).

## 4. Discussion

The results of TCGA database analysis showed that the expression of B2M was increased in most tumors and decreased in a few tumors (Figure 1). Josson et al. reported that overexpression of B2M promotes the growth and progression of renal cell carcinoma, lung cancer, prostate cancer, and breast cancer [19]. Some researchers compared the preoperative serum B2M concentration of 40 patients with renal cell carcinoma and 23 normal controls and found that the preoperative serum B2M level increased in 70% of renal cell carcinoma patients [20]. Since then, researchers have demonstrated that B2M can promote the growth of human renal cell carcinoma [21] by activating the protein kinase A, cyclic adenosine monophosphate response element binding protein, and vascular endothelial growth factor axis. At the same time, a large number of studies have found that serum B2M levels in lung cancer [22, 23], prostate cancer [24–27], breast cancer [28, 29], and hematological malignancies have also increased [30–32]. We downloaded 41 samples of normal tissue adjacent to cancer and 286 samples of colon cancer from TCGA database. The results showed that the expression of B2M gene in colon cancer tissues was significantly lower than that in adjacent normal tissues.

The article "Analysis of the B2M Expression in Colon Adenocarcinoma and Its Correlation with Patient Prognosis" was retracted in 2023. Reasons: suspected computer-generated content; unreliable results or conclusions; lack of ethics approval or compliance; missing or withdrawn patient consent.

DNA methylation status of the CpG island is often related to the transcriptional silence of related genes [33, 34]. Some researchers believe that DNA methylation plays a role in regulating HLA class I antigen presentation [35]. At present, there are only a few studies on the methylation status of tumor B2M gene. Gyorffy et al. found that epigenetic hypermethylation can cause loss or downregulation of HLAs and B2M expression in breast cancer [36]. At the same time, some researchers believe that hypermethylation of the B2M gene promoter may affect the antigen presentation of HLA class I molecules, which may lead to immune escape and immunotherapy resistance of colorectal cancer [37]. In addition, Cornelia et al. found that elimination of DNA methylation by DNMT inhibitors upregulated the expression of B2M at RNA and protein levels [38] in colon adenocarcinoma. However, the analysis of TCGA database showed that the methylation level of B2M gene promoter in colon adenocarcinoma tissues was lower than that in adjacent normal tissues. At the same time, the methylation of B2M gene promoter was at a very low level in both adjacent normal tissues and colon cancer tissues. This suggests that the low expression of B2M in colon cancer tissues may not be caused by methylation of the B2M gene promoter, but by B2M gene mutation [39, 40].

B2M is an important subunit of MHC class I molecules, which plays an antitumor role by promoting MHC class I molecules-mediated tumor antigen presentation and T cell recognition [2]. Therefore, we believe that B2M gene is a tumor suppressor gene in colon cancer, and its low expression in colon cancer tissue can promote the occurrence and development of colon cancer. We then analyzed the expression of B2M in different stages of colon cancer by TCGA database. The results showed that the expression level of B2M mRNA decreased with the progression of colon cancer stage, and the expression levels of B2M mRNA were different between stages I and IV, II and IV. In addition, we can also see that the expression level of B2M mRNA is different between colon adenocarcinoma and mucinous adenocarcinoma. The expression of B2M mRNA in colonic mucinous adenocarcinoma was higher than that in colonic adenocarcinoma.

TP53 is a common tumor suppressor gene, which plays a role in a variety of tumors. Mutations of TP53 are the most common in human tumors and are often associated with poor prognosis [41]. The missense mutation of TP53 is very common in human cancers, which can lead to the inactivation of the tumor suppressive effect of mutant p53 protein, which is conducive to the proliferation and survival of cancer cells, thus promoting tumor invasion, migration and chemotherapy resistance [42, 43]. The frequency of TP53 mutation in colorectal cancer ranged from 40% to 50% [44]. Through TCGA database analysis, we found that the expression level of B2M in colon cancer tissues with TP53 mutation was lower than that without mutation. It is suggested that the low expression of B2M in colon cancer is related to TP53 gene mutation. The expression level of B2M in colon cancer tissues with TP53 mutation is lower, and the tumor is easier to metastasize and more aggressive.

The article "Analysis of the B2M Expression in Colon Adenocarcinoma and Its Correlation with Patient Prognosis" was retracted in 2023. Reasons: suspected computer-generated content; unreliable results or conclusions; lack of ethics approval or compliance; missing or withdrawn patient consent.

In addition, we also found that the expression level of B2M gene had racial difference, but it was not related to gender, age and weight of patients with colon cancer.

The effect of B2M expression level on the prognosis of cancer patients is different. The high expression of B2M gene is associated with poor prognosis in most cancer patients. It has been reported that elevated B2M can worsen the prognosis of patients with renal cell carcinoma [45], prostate cancer, breast cancer [29], hematological malignancy [30, 31, 46–48] and glioma [49]. At the same time, Kloor et al. thought that the B2M mutation was associated with reduced metastasis and recurrence of colon cancer [40, 50, 51]. However, Shrout and Bianchini et al. found that the low expression of B2M was associated with lymph node metastasis and poor prognosis in patients with colorectal cancer [52, 53]. However, we found that the expression level of B2M was not related to the status of lymph node metastasis in patients with colon cancer through TCGA database analysis, which was inconsistent with the results reported in the literature. This may be because the TCGA database analyses tumor metastasis in axillary lymph nodes, while regional lymph node metastasis is the most common in colon cancer. At the same time, different researchers have drawn different conclusions on the impact of B2M expression level on lymph node metastasis and prognosis of colon cancer, so it is necessary to strengthen further research in this area.

To sum up, B2M may be a potential tumor suppressor gene in colon cancer. The decreased expression of B2M after mutation can cause immune escape of colon cancer cells, thus affecting the therapeutic effect and prognosis. However, there are still some contradictions about the role of B2M in colon cancer. Therefore, more research is needed to continue to explore the role of B2M in colon adenocarcinoma.

The article "Analysis of the B2M Expression in Colon Adenocarcinoma and Its Correlation with Patient Prognosis" was retracted in 2023. Reasons: suspected computer-generated content; unreliable results or conclusions; lack of ethics approval or compliance; missing or withdrawn patient consent.

## Figures and Tables

**Figure 1:** Expression of the B2M gene in the tumor tissues of the TCGA database.

**Figure 2:** Expression of B2M in COAD based on sample types.

**Figure 3:** Promoter methylation level of B2M in COAD.

**Figure 4:** Expression of B2M in COAD based on individual cancer stages.

**Figure 5:** Expression of B2M in COAD based on histological subtypes.

**Figure 6:** Expression of B2M in COAD based on nodal metastasis status.

**Figure 7:** Expression of B2M in COAD based on TP53 mutation status.

**Figure 8:** Expression of B2M in COAD based on patient's gender.

**Figure 9:** Expression of B2M in COAD based on patient's age.

**Figure 10:** Expression of B2M in COAD based on patient's weight.

**Figure 11:** Expression of B2M in COAD based on patient's race.

**Figure 12:** Effect of B2M expression level on COAD patient survival.

**Figure 13:** Genes positively correlated with B2M in COAD.

**Figure 14:** Genes negatively correlated with B2M in COAD.

**Table 1:** The clinical characteristics of the COAD patients in the TCGA.

Clinical features	Classification	Percentage (%)
Gender, *n* (%)	Male	156 (55.1%)
	Female	127 (44.9%)

Age, *n* (%)	21∼60	102 (36.0%)
	61∼100	181 (64.0%)

Weight, *n* (%)	Normal weight (BMI: 18.5∼25)	70 (33.3%)
	Extreme weight (BMI: 25∼30)	74 (35.2%)
	Obese (BMI: 30∼40)	56 (26.7%)
	Extreme Obese (BMI > 40)	10 (4.8%)

Clinical stage, *n* (%)	Stage I	45 (16.4%)
	Stage II	110 (40.2%)
	Stage III	80 (29.2%)
	Stage IV	39 (14.2%)

Histological subtypes, *n* (%)	Adenocarcinoma	243 (86.8%)
	Mucinous adenocarcinoma	37 (13.2%)

## Data Availability

The data used and/or analyzed during the current study are available from the corresponding author upon request.
